The article "Differential expression of the angiogenesis growth factors in psoriasis vulgaris" was published in 2012. Journal: BMC Res Notes.

# Differential expression of the angiogenesis growth factors in psoriasis vulgaris

**DOI:** 10.1186/1756-0500-5-201

**Published:** 2012-07-03

**Authors:** Siaw-Cheok Liew, Esha Das-Gupta, Srikumar Chakravarthi, Shew-Fung Wong, Nagarajah Lee, Najeeb Safdar, Adawiyah Jamil

**Affiliations:** 1 Department of Postgraduate Studies and Research, International Medical University, Kuala Lumpur, Malaysia; 2 Department of Internal Medicine, International Medical University, Seremban, Malaysia; 3 Open University, Kuala Lumpur, Malaysia; 4 Department of Dermatology, Tuanku Ja’afar Hospital, Seremban, Malaysia; 5 Department of Dermatology, Kuala Lumpur Hospital, Kuala Lumpur, Malaysia

## Abstract

**Background:**

Angiogenesis has been reported to be one of the contributory factors to the pathogenesis of psoriasis vulgaris. This study aims to compare the expression of different angiogenesis growth factors namely (1) the vascular endothelial growth factor (VEGF) subfamily: A, B, C, D and placenta growth factor (PlGF); (2) nerve growth factor (NGF) and (3) von Willebrand factor (vWFr) in the skins of patients with psoriasis vulgaris and non-psoriatic volunteers.

**Results:**

Comparative immunohistochemistry study was performed on the paraffin-sectioned psoriatic and healthy skins with the abovementioned markers. VEGF-C (*p* = 0.016) and NGF (*p* = 0.027) were expressed intensely in the cases when compared with the controls. The NGF was the only marker that was solely expressed in the cases and absent in all the controls.

**Conclusion:**

The NGF (angiogenesis) and VEGF-C (lymphangiogenesis) might play a crucial role in the pathogenesis of psoriasis vulgaris and could be researched further as potential new targeted therapies for psoriasis vulgaris.

## Background

Angiogenesis or neovascularization refers to the formation of new capillary vessels from the existing vascular bed [1]. Angiogenesis was first reported in 1972 as a contributory factor in the pathogenesis of psoriasis vulgaris, replacing the initial reports of the disease being purely immunologic in nature [2]. Psoriasis has been studied in the light of it being angiogenic in nature since then [3]. Four-fold increase of endothelial microvascular bed was seen in the psoriatic skin but not in normal skin, thus signifying the importance of angiogenesis in psoriasis [4]. Dermal microvascular expansion with abnormal orientation and dilatation of capillaries in the biopsies of the psoriatic skin revealed that the disease was angiogenesis dependent [5]. Other supporting evidences include the increased of blood flow observed in the skin biopsy peripheral to the psoriatic lesion that was obtained with laser doppler fluxmetry [6], the increased of the microvasculature of the lesion seen in audioradiograph [7] and the elongated capillary loops in psoriasis as reported in an ultra-structural study [8].

The article "Differential expression of the angiogenesis growth factors in psoriasis vulgaris" was published in 2012. Journal: BMC Res Notes.

The keratinocytes in the psoriatic skin lesions were recognized as a source of pro-angiogenic cytokines which induce angiogenesis, namely the vascular endothelial growth factor (VEGF). Other commonly recognized cytokines were endothelial cell stimulating angiogenesis factor (ESAF), tumour necrosis factor-α (TNF-α) and platelet derived growth factors (PDGF) [9-14].

The VEGF-A has four isoforms - (VEGF_121_, VEGF_165_, VEGF_189_ and VEGF_206_) [9,15] and was structurally related to the VEGF-B, VEGF-C, VEGF-D and placenta growth factor (PlGF) [16]. The role of VEGF-A, formally known as VEGF, in angiogenesis was well established [17-19]. The VEGF-A regulates the growth of the vascular endothelial cells of the arteries, veins and the lymphatics [20]. The VEGF-A was involved in vasculogenesis and angiogenesis during the embryonic and early postnatal development [20-22], skeletal growth [23], wound healing [24-26] and ovarian angiogenesis [27-29]. Up-regulation of the VEGF-A mRNA expression was reported in tumours of the lung [30], thyroid [31], breast [32], liver [33], kidney and bladder [34] and the female reproductive tracts [35,36]. The VEGF-A has been associated with skin inflammation and pathogenesis of psoriasis [17,37]. The keratinocytes of the psoriatic skin expressed the VEGF-A receptors 1 and 2 on their surfaces. The VEGF-A secreted by the keratinocytes was able to bind to these receptors and activate the signaling pathway via an autocrine manner [38,39]. The VEGF-A expression at the basal keratinocytes showed psoriatic-like skin inflammation with increased tortousity and branching of dermal blood vessels in a mouse model [40,41].

The VEGF-B (188 amino acids) was found abundantly in muscle and myocardium. The VEGF-B stimulated the growth of the vascular endothelial cells and involved in embryogenic angiogenesis [42,43]. The VEGF-C (399 amino acids) stimulated the growth of human lung endothelial cells and was involved in lymphangiogenesis [44,45]. Similar to VEGF-C, VEGF-D is lymphangiogenic in nature [46,47]. The placenta growth factor (PlGF) was expressed during ischaemia, inflammation, wound healing and tumorigenesis [48,49]. Though the VEGF-A has been well-associated in the pathogenesis of psoriasis, the structurally related subfamily (VEGF-B, C, D and PlGF) immunohistochemistry expression in psoriasis is still unknown. Differential immunohistochemistry expression of these subfamily molecules with the VEGF-A is not documented previously.

The NGF was identified as a novel angiogenic molecule, be it in the physiological (wound healing) [50] or pathological conditions (ischaemia and tumour growth) [51-53]. The NGF was highly expressed in blood vessels of hypertensive rats [54], hearts of ischaemic rats [55] and brains of hypertensive rats [56]. The von Willebrand factor (vWFr) was involved in the endothelial cell activation which leads to tumours angiogenesis [57].

The article "Differential expression of the angiogenesis growth factors in psoriasis vulgaris" was published in 2012. Journal: BMC Res Notes.

This study aims to investigate the immunohistochemistry expression of the vascular endothelial growth factor (VEGF-A) in comparison with its subfamily i.e. VEGF-B, C, D and PlGF, and also with the recently identified angiogenesis growth factors (NGF and vWFr) in the cases and controls. The comparative levels of immunohistochemistry expression of the VEGF (subfamily A, B, C, D and PlGF), NGF and vWFr in psoriasis vulgaris are still unknown. We investigated the expression of these angiogenesis growth factors in psoriasis vulgaris patients and healthy controls. The association of these angiogenesis growth factors with the pathogenesis of psoriasis vulgaris will be of great importance in the understanding of the nature and progression of the disease and also for therapeutic purposes.

## Methods

### Study population

The cases for this retrospective study were recruited from the Dermatology Department of Hospital Kuala Lumpur, Kuala Lumpur and Tuanku Ja’afar Hospital, Seremban, Malaysia. All the patients with psoriasis vulgaris (n = 17) were clinically examined and diagnosed by the dermatologist. Healthy controls (n = 6) were recruited from the Orthopaedic Department of Tuanku Ja’afar Hospital, Seremban. The cases and controls were well-informed about the nature of this study and the participations were voluntary. Informed consent was obtained from each of the participants. The cases were psoriasis vulgaris patients that were not receiving any form of systemic or phototherapy. Topical therapy had been discontinued for 2 weeks prior to the procedures of obtaining the biopsies. Only topical emollients were used. A 6 mm punch biopsy was obtained from each subject and fixed in 10% buffered formalin solution. The protocol of this study was designed according to the Declaration of Helsinki and was approved by the ethics committee of our University. The characteristics of the cases and controls are summarized in Table 1.

**Table 1:** Characteristics of Study Population

	**Cases** **(n = 17**)	**Controls** **(n = 6)**
**Age**, mean ± SD	47.94 ± 10.55	42.33 ± 22.38
**Gender**		
Male, n (%)	10 (59%)	4 (67%)
Female, n (%)	7 (41%)	2 (33%)
**Race**		
Chinese, n (%)	4 (24%)	1 (17%)
Indian, n (%)	4 (24%)	1 (17%)
Malay, n (%)	9 (52%)	4 (66%)
**PASI**, mean ± SD	7.25 ± 4.78	N/A
**Smoking,** n (%)	2 (11.8%)	0 (0)
**BMI**	25.94 ± 4.80	20.6 ± 2.69
**Additional Co-morbidities** (SLE, Chron’s, Ulcerative colitis, Rheumatoid Arthritis).	NIL	NIL

The article "Differential expression of the angiogenesis growth factors in psoriasis vulgaris" was published in 2012. Journal: BMC Res Notes.

### Immunohistochemistry

The fixed biopsies were processed, embedded in paraffin and sectioned at 4 μm with a microtome (Leica RM 2135, Germany). The sections were placed on poly-L-lysine coated slides and were incubated at 60°C for 30 minutes for proper adherence and drying. The sections were deparraffinized by subjecting to 3 changes of xylene substitute (Sigma, USA) for 3 minutes each. The sections were rehydrated in descending concentration of alcohols gradually from 100% to 20% and lastly in water (3 minutes each). Antigen retrieval procedure was performed using a microwave in citrate buffer (pH 6.0) for 15 minutes. The non-specific areas of the sections were blocked with blocking solution (1: 10; Kirkegaard & Perry Lab (KPL), Maryland USA) for 4 minutes and followed by swine normal serum (1: 20; Dako Cytomation, Denmark). The sections were either incubated with rabbit anti-VEGF-A (polyclonal; 1: 25; Millipore, CA, USA), mouse anti-VEGF-B (monoclonal; 1: 25; Abcam, Camb, UK), rabbit anti-VEGF-C (polyclonal; 1: 25; Abcam, Camb, UK), rabbit anti-VEGF-D (polyclonal; 1: 25; Abcam, Camb, UK), rabbit anti-NGF (polyclonal; 1: 25; Abcam, Camb, UK), rabbit anti-PlGF (polyclonal; 1: 25; Abcam, Camb, UK) and rabbit anti-vWFr (polyclonal; 1: 25; Abcam, Camb, UK) overnight at 4°C in a wet chamber respectively. After the incubation, the slides were washed with phosphate buffered saline (PBS) for 10 minutes before incubation with horseradish peroxidase conjugated anti-mouse or anti-rabbit immunoglobulins (1: 200) respectively for 2 hours at room temperature. The slides were washed with PBS for 10 minutes and incubated with TrueBlue peroxidase substrate (KPL, Maryland USA) for 10 minutes. The substrate was washed away with ultra-pure water for 3 minutes and the samples were counterstained with KPL Orcein for 3 minutes. The slides were then rinsed with ultra-pure water, dehydrated in ascending concentration of alcohols every 3 minutes, dried, mounted with Depex and observed under a compound microscope (Nikon, Japan) at 40X, 100X, 200X and 400X magnifications. The intensity of the staining was scored: negative, weak, moderate and strong. The scores were 0 for negative, 1 for weak, 2 for moderate and 3 for strong staining patterns. The mean score for each growth factor was calculated.

### Statistical analysis

An Independent *T*-test and subsequent Mann–Whitney-*U* test were used to analyze the staining scoring of these markers on cases and controls. Pearson’s correlation was used to determine the correlation of the Psoriatic Area and Severity Index (PASI) with the intensity of the staining for each marker. P values of less than 0.05 were considered statistically significant.

The article "Differential expression of the angiogenesis growth factors in psoriasis vulgaris" was published in 2012. Journal: BMC Res Notes.

## Results

### PASI classification

The average PASI score for the cases was 7.247 ± 4.780. The age (mean) for the cases was 47.94 years and for the controls was 42.33 years.

### Immunohistochemistry

The mean scores (± standard deviation) for VEGF-A, VEGF-B, VEGF-C, VEGF-D, NGF, PlGF and vWFr immunoreactivities in cases were 1.76 ± 1.03, 0.00, 1.59 ± 1.12, 0.35 ± 0.61, 1.24 ± 1.25, 1.12 ± 1.32 and 0.65 ± 1.06 respectively (Figure 1). The mean scores (± standard deviation) for VEGF-A, VEGF-B, VEGF-C, VEGF-D, NGF, PlGF and vWFr staining in controls were 1.83 ± 0.98, 0.00, 0.33 ± 0.52, 0.33 ± 0.52, 0.00, 0.33 ± 0.82 and 1.67 ± 0.52 respectively (Figure 2). The immunohistochemistry staining of the abovementioned markers on psoriasis vulgaris skin were shown in Figure 3.

**Figure 1:** The mean angiogenesis markers staining score for cases (n = 17).

**Figure 2:** The mean angiogenesis markers staining score for controls (n = 6).

**Figure 3:** **Immunohistochemistry staining of the skins of patients with psoriasis vulgaris.** (**A**) Strong VEGF-A expression in the epidermis and dermis of the psoriatic skin at 200 x magnification. (**B**) No staining of VEGF-B in all layers of the psoriatic skin at 200 x magnification. (**C**) Strong staining of VEGF-C in the dermal layer of the psoriatic skin at 200 x magnification. (**D**) Moderate staining of VEGF-D in dermal layer of the psoriatic skin at 100 x magnification. (**E**) Moderate staining of PlGF in all layers of the psoriatic skin at 200 x magnification. (**F**) Strong staining of NGF in dermal layer of psoriatic skin at 200 x magnification. (**G**) Weak staining of vWFR in the epidermis of the psoriatic skin at 200 x magnification. Note: blue to purple indicated positive immunoreactivities with red as counterstain. (**H**) Haematoxylin and eosin (**H**&**E**) staining of the psoriatic skin at 200 x magnification.

There was no significant correlation between the expression of these growth factors with PASI scores: VEGF-A (*p* = 0.399), VEGF-B (negative staining for cases and controls), VEGF-C (*p* = 0.232), VEGF-D (*p* = 0.216), NGF (*p* = 0.177), PlGF (*p* = 0.404) and vWFr (*p* = 0.169).

An Independent *T*-test and subsequent Mann Whitney *U* test were performed for multiple comparisons between the expression of these markers, cases and controls. The intensity of staining VEGF-C (*p* = 0.016) was significantly higher in the cases when compared with the controls. Mann Whitney *U* test showed similar result (*p* = 0.016). Significant intensity in expression of the NGF was observed in cases compared with controls (*p* = 0.027, Independent *T*-test; *p* = 0.020, Mann Whitney *U* test). The other growth factors did not show any significant differences in the intensities of their staining between cases and controls. The VEGF-A (*p* = 0.889), VEGF-B (negative staining for cases and controls), VEGF-D (*p* = 0.945), PlGF (*p* = 0.189) and interestingly vWFr were significantly expressed in the controls instead of the cases (*p* = 0.036).

The article "Differential expression of the angiogenesis growth factors in psoriasis vulgaris" was published in 2012. Journal: BMC Res Notes.

### Homocysteine and angiogenesis markers

The mean homocysteine level in the cases was 16.41 ± 3.90 μmol/L. No statistically significant correlation between these markers and homocysteine levels in cases: VEGF-A (*p* = 0.853), VEGF-B (negative staining for cases and controls), VEGF-C (*p* = 0.139), VEGF-D (*p* = 0.637), NGF (*p* = 0.374), PlGF (*p* = 0.795) and vWFr (*p* = 0.152).

## Discussion

Cutaneous angiogenesis occurs during the normal physiological stages of hair growth [58] and so could angiogenesis be found in pathological cutaneous conditions such as malignant melanoma [59] and psoriasis [60]. Epidermal keratinocytes have been identified mainly as the source of the VEGF, PlGF, NGF and vWFR that contribute to psoriasis angiogenesis. The VEGF-C and VEGF-D are expressed by the lymphatic endothelium contributing to lymphangiogenesis [61]. The VEGF-A has been well-established as an angiogenesis factor in psoriasis vulgaris but the comparative expressions of its subfamily i.e. the VEGF-B, VEGF-C, VEGF-D and PlGF with VEGF-A were lacking. The newly discovered angiogenesis growth factors’ (NGF and vWFr) expression in psoriasis vulgaris in comparison with the VEGF family has never been documented.

No significant difference in the expression of VEGF-A (*p* = 0.889) between the cases and controls was observed. The VEGF-A was expressed in the keratinocytes of the skins in the cases and was expressed in the dermal layer of the skins in the controls. In the cases, the VEGF-A was expressed in the keratinocytes of the epidermis and some fibroblasts of the dermal layer. Henno et al. [62,63] reported in both these studies, the expression of VEGF-A mRNA was significantly increased in the psoriasis patients when compared to the controls. Bhushan *et al*. [64] reported that VEGF is produced predominantly by the keratinocytes, far lesser extent by the fibroblast. Creamer *et al*. [65] reported that the VEGF-A enhances vascular permeability in eczema patients in response to inflammation. Therefore, the increase of the expression of the VEGF in the controls could be due to the inflammatory process subsequent to orthopaedic trauma.

The article "Differential expression of the angiogenesis growth factors in psoriasis vulgaris" was published in 2012. Journal: BMC Res Notes.

The NGF was significantly expressed (*p* = 0.027) solely in the skin of the psoriatic patients compared with healthy controls in the present study. Similar finding was reported by Raychaudhuri *et al.*[66] who compared the expression of the NGF in psoriasis vulgaris and lichen planus in human. Fantini *et al*. [67] reported tissue extracts obtained from psoriasis vulgaris patients showed higher levels of the NGF compared with healthy controls. The role of NGF on the development of psoriasis is still poorly understood though related to neurogenic inflammatory nature of the NGF postulation [66]. The NGF is a pleiotropic factor acting both on the neuronal and vascular levels [68]. Therefore, angiogenic nature of the NGF could have contributed to the high levels of the NGF seen in the psoriatic skin compared with the controls. The significant association between the NGF expression and psoriasis in comparison to the other angiogenesis growth factors investigated in this study may suggest the potential use of the NGF as an indicator for the development of psoriasis vulgaris. Unlike the VEGF-A, the expression of nerve growth factor was very specific in psoriatic skin. Therefore, would a new targeted therapy for the NGF be the future research area for psoriasis vulgaris?

In this study we also found that the VEGF-C intensity of staining were significantly (*p* = 0.016) higher in the psoriatic skin compared with the normal skin. Henno et al. [62,63] reported the significant expression of mRNA in the cases compared to the controls. The VEGF-C expression revealed the role of lymphangiogenesis in psoriasis vulgaris. Lazarovici *et al.* in his article “cross talk between NGF and VEGF” stated expression of the NGF and the VEGF resulted in the activation of two common intracellular signaling cascades, trkA for the NGF and VEGFR-2 for the VEGF in endothelial cells that were involved in the proliferation and survival of these cells. Therefore, there was a probability of the concerting effects of the NGF and VEGF in controlling angiogenesis processes [69]. Perhaps, the same theoretical principle could also be researched further on the synergistic interplay between the NGF and the VEGF-C. A new drug discovery study would probably target both the VEGF-C and NGF activities.

Another interesting finding would be the significant higher intensity of staining of the VEGF-C (*p* = 0.016) in the psoriasis vulgaris skin compared with the controls, but not for the VEGF-D (*p* = 0.945) although both are lymphangiogenesis in nature and closely related structurally [42]. Perhaps similar to previous speculation, the discrepancies in the results could be due to the different tissue distribution, i.e. the VEGF-C found mainly in heart, placenta, ovary and small intestine whereas the VEGF-D was commonly found in the lungs. Otherwise, could there be another lymphangiogenesis receptor specific to the VEGF-C cutaneously that was not receptive for the VEGF-D unlike the conventional Flt-4 receptor that was shared between the two?

The article "Differential expression of the angiogenesis growth factors in psoriasis vulgaris" was published in 2012. Journal: BMC Res Notes.

## Conclusion

In conclusion, this study involved a small sample size and showed a significant finding on the contribution of the NGF and the VEGF-C in the pathogenesis of psoriasis vulgaris. A bigger pool of samples could be used in future to look at the association of NGF with psoriasis vulgaris and to research further on the angiogenesis pathways of NGF on psoriasis vulgaris. The same may also be investigated for the VEGF-C. The interplay of the NGF and the VEGF-C could also be investigated and the expansion of knowledge in the synergistic interplay pathway of the NGF and VEGF-C in the angiogenic pathogenesis of psoriasis vulgaris would prove useful for the development of future therapeutic agent against the signaling cascades mediated by the NGF and VEGF-C.

## Competing Interests

The authors declare that they have no competing interests.

## Authors Contributions

SCL: participated in the conception of the study, the inception of the study design, carried out the patients sampling, immunohistochemistry staining, reviewing of the slides and drafting of the manuscript. EDG, NS, AJ: participated in the conception of the study, the inception of the study design, carried out the patients sampling and drafting of the manuscript. SC and SFW: participated in the conception of the study, the inception of the study design, immunohistochemistry staining, reviewing of the slides and drafting of the manuscript. N Lee participated in the conception of the study, the inception of the study design and performed and advised on the statistical analysis. All authors read and approved the final manuscript.
